# Application of the Truncated Zero-Inflated Double Poisson for Determining of the Effecting Factors on the Number of Coronary Artery Stenosis

**DOI:** 10.1155/2022/5353539

**Published:** 2022-01-13

**Authors:** Arezoo Orooji, Toktam Sahranavard, Mohammad-Taghi Shakeri, Mohammad Tajfard, Seyed Ehsan Saffari

**Affiliations:** ^1^Department of Epidemiology and Biostatistics, Faculty of Health Sciences, Mashhad University of Medical Sciences, Mashhad, Iran; ^2^Faculty of Medicine, Mashhad University of Medical Science, Mashhad, Iran; ^3^Department of Epidemiology & Biostatistics, MUMS, Mashhad, Iran; ^4^Department of Health Education and Health Promotion, Faculty of Health, Mashhad University of Medical Sciences, Mashhad, Iran; ^5^Social Determinants of Health Research Center, Mashhad University of Medical Sciences, Mashhad, Iran; ^6^Centre for Quantitative Medicine, Duke-NUS Medical School, National University of Singapore, Singapore

## Abstract

**Background:**

Risk factors of coronary heart disease have been discussed in the literature; however, conventional statistical models are not appropriate when the outcome of interest is number of vessels with obstructive coronary artery disease. In this paper, a novel statistical model is discussed to investigate the risk factors of number of vessels with obstructive coronary artery disease.

**Methods:**

This cross-sectional study was conducted on 633 elderly cardiovascular patients at Ghaem Hospital, Mashhad, Iran from September 2011 to May 2013. Clinical outcome is number of vessels with obstructive coronary artery disease (=0, 1, 2, 3), and predictor variables are baseline demographics and clinical features. A right-truncated zero-inflated double Poisson regression model is performed which can accommodate both underdispersion and excess zeros in the outcome. The goodness-of-fit of the proposed model is compared with conventional regression models.

**Results:**

Out of 633 cardiovascular patients, 327 were male (51.7%). Mean age was ~65 ± 7 years (for individuals with zero, one ,and two coronary artery stenosis) and ~66 ± 7 years (for individuals with three coronary artery stenosis). BMI (0.04 ± 0.01, *p* = 0.011) and female gender (0.19 ± 0.09, *p* = 0.032) were significant associated with the count part of the model, and only BMI (−0.47 ± 0.2, *p* = 0.011) was significantly predictive of logit part of the model. The goodness-of-fit measurements indicate that the proposed model outperforms the conventional regression models.

**Conclusion:**

The proposal regression model shows a better fit compared to the standard regression analysis in modeling number of vessels with obstructive coronary artery disease. Hence, using truncated zero-inflated double Poisson regression model—as an alternative model—is advised to study the risk factors of number of involved vessels of coronary artery stenosis.

## 1. Background

The cause of one out of three deaths is cardiovascular disease [1]. It is noted that coronary heart disease is one of the two highest causes of mortality in Australia and UK [2]. Coronary heart disease is the most common reason of disability with 13.3% of deaths worldwide [3]. Coronary artery disease develops when the major blood vessels—that supply heart with blood, oxygen, and nutrients (coronary arteries)—become damaged or narrowed. The narrowing may lead to ischemic heart disease and even death [4]. Coronary angiography is the gold standard diagnostic method for coronary heart disease and an expensive approach in terms of cost and having several side effects [5]. Prognostic factors of coronary heart disease have been discussed in the literature, including gender, age, smoking status, diabetes mellitus, systemic hypertension, hypercholesterolemia, high sensitivity C reactive protein (hs-CRP), and body mass index (BMI) [3, 6–8].

Regression models are commonly used to investigate the association between independent variables and clinical outcome [9]. If the clinical outcome is a count variable, count regression models are recommended. In many clinical data, there is a high proportion of zeros in the outcome—excess zeros. Zero-inflated (ZI) count models are typically used to model such data. In ZI models, a mixture of two separate data generation processes is performed: one generates only zeros, and the other is a count distribution data-generating process. Determining which of the processes leads to observation is done by a Bernoulli experiment. In addition, there are two types of zeros in such data: structural zeros (or true zeros) which refers to a not-at-risk situation for a behavior of interest and random zeros (or false zeros) which refers to an at-risk situation due to sampling variability. The mixture distribution discussed above is one way of accommodating the difference between structural and random zeros [10–12].

In many applications, there are some extreme values at the right side of the distribution which causes overdispersion (variance is greater than mean). One solution to overcome this problem is to truncate the extreme values above a specific point. On the other hand, there are situations where the outcome of interest is right-truncated by definition. An example of this scenario is number of vessels with obstructive coronary artery disease which is limited to a maximum of 3 vessels. If the conventional count regression models (with no truncation) are performed on number of involved vessels with obstructive coronary artery disease, predicted probabilities will be generated for all nonnegative values for number of involved vessels which is not meaningful [13, 14] . Hence, a right-truncated model seems to be a good approach.

Poisson regression is the most common approach used for modeling count response variables [11, 14]. Mean is assumed to be equal to variance in the Poisson regression model; hence, this model cannot perform well when under and overdispersion scenarios [13]. Overdispersion has been addressed pretty well in literature; however, models which can accommodate underdispersion are limited [11–13]. Number of involved vessels in coronary artery stenosis is an underdispersed outcome in our case study.

The aim of this study is to introduce zero-inflated double Poisson (ZIDP) model with right truncation as an alternative novel approach addressing both excess zeros and underdispersion problems simultaneously for patient with coronary artery stenosis. Validation of this model will be assessed via comparison of the goodness-of-fit measurements (including -2LogLikelihood (-2LL) and Akaike information criterion (AIC)) of the proposed model with other alternative count regression models.

## 2. Methods

### 2.1. Data Description

This cross-sectional study was conducted on 633 cardiovascular patients who visited cardiovascular department and received catheter angiography at Ghaem Hospital, Mashhad, Iran, from September 2011 to May 2013. Inclusion criteria were aged >55 years old (as the intention was to target a potentially sicker population) [15–19], and exclusion criteria were pregnant and lactating women and individuals with rheumatic disease, chronic liver disease, kidney disease, any type of cancer, infectious diseases in the last 3 months, history of any surgery in the last 3 months, history of coronary angioplasty, immunological disease, any disease associated with inflammatory bowel disease, and those taking any of the following medications: steroids, penicillin, oral contraceptives, or hormone replacement therapy.

The outcome variable is number of vessels involved in coronary artery stenosis revealed by angiography. Predictor variables included are the known risk factors of coronary artery disease which are available in this study including gender, age, body mass index (BMI), history of smoking, hypertension history, diabetic history, hyperlipidemia history, cardiovascular diseases history, and myocardial infarction history [20, 21].

### 2.2. Data Analysis and Statistical Methods

The clinical outcome of this study is nonnegative integer value (= 0, 1, 2, 3). Demographics and clinical features were reported as mean ± standard deviation and frequency (percent) for continuous and categorical parameters, respectively, and compared by the number of involved vessels of coronary artery stenosis. Various count regression models were conducted to investigate the association between the number of coronary artery stenosis and the above parameters, including Poisson and negative binomial regression models (as the most commonly used models), zero-inflated Poisson (ZIP) and zero-inflated negative binomial (ZINB) models (due to high proportion of zeros), and right-truncated ZIP and ZINB models (since the number of coronary artery stenosis is ≤3). Finally, a right-truncated zero-inflated double Poisson is performed which can accommodate both underdispersion and excess zeros in the outcome. Parameter estimates were obtained using maximum likelihood approach. Goodness-of-fit measures—including -2LogLikelihood and Akaike information criterion—were calculated for each model to assess the validation of the proposed model. Statistical significance was set at *p* < 0.05. Statistical analyses were performed using SAS software version 9.4 for Windows (SAS, Inc., Cary, NC).

#### 2.2.1. Double Poisson Regression

Double Poisson regression suggested by Efron (1986) is a count model which can be used for over- and underdispersed data, where variance is greater or less than mean, respectively [22]. This model incorporates a dispersion parameter to handle over- and underdispersion. The probability mass function of a double Poisson distribution is given by

(1) $$\begin{array}{c} P\left(Y=y\right)=f\mu \varphi \left(y\right)=c\left(\mu \varphi \right)\left(\varphi \frac{1}{2}e^{-\varphi \mu }\right)\left(\frac{e^{-y}y^{y}}{y!}\right){\left(\frac{e\mu }{y}\right)}^{jy},y=0,1,2,\cdots , \end{array}$$

where *c*(*μ*, *φ*) is a constant and given by

(2) $$\begin{array}{c} \frac{1}{c\left(\mu ,\varphi \right)}=\overset{\infty }{\underset{y=0}{\sum }}f_{\mu ,\varphi }\left(y\right)\approx 1+\frac{1‐\varphi }{12\mu \varphi }\left(1+\frac{1}{\mu \varphi }\right), \end{array}$$

ensuring the probability mass function is perforce normalized to sum to unity in most cases. *μ* and *ϕ* are the mean and dispersion parameters. The link function is defined as *μ* = exp(*xβ*), where *x* is a vector of covariates associated with *Y*, and *β* is a vector of unknown regression coefficients. The expected value and variance of the exact density are approximated by *μ* and *μ*/*ϕ*. Hence, double Poisson allows for both underdispersion (*ϕ* > 1) and overdispersion (*ϕ* < 1). The double Poisson model collapse to Poisson model when *ϕ* = 1.

#### 2.2.2. Excess Zero with Right Truncation

There are situations where high proportion of zeros is available in count data. Mixture models such as zero-inflated models can handle the excess zeros in the outcome variable. In this study, there is excess zeros in number of coronary artery stenosis. The probability mass function of ZIDP model is given by

(3) $$\begin{array}{c} p\left(Y=y\right)=\left\{\begin{array}{c} \pi +\left(1‐\pi \right)c\left(\mu ,\varphi \right)\left(\varphi^{\frac{1}{2}}e^{‐\varphi \mu }\right),y=0,\\ \left(1‐\pi \right)c\left(\mu ,\varphi \right)\left(\varphi^{\frac{1}{2}}{\text{e}}^{‐\varphi \mu }\right){\left(\frac{e^{-y}y^{y}}{y!}\right)}^{\varphi \text{y}},y>0, \end{array}\right. \end{array}$$

where *π* is a link function defined as exp(*xβ*)/1 + exp(*xβ*).

Since the number of coronary artery stenosis in cardiovascular disease cannot be more than three, a right-truncated approach is applied on the ZIDP model. Therefore, probability mass function for truncated zero-inflated double Poisson (TZIDP) is given by

(4) $$\begin{array}{c} p\left(Y=y\right)=\left\{\begin{array}{c} \frac{\pi +\left(1‐\pi \right)c\left(\mu ,\varphi \right)\left(\varphi^{1/2}e^{‐\varphi \mu }\right)}{1‐\sum_{y=4}^{\infty }\left(1‐\pi \right)c\left(\mu ,\varphi \right)\left(\varphi^{1/2}e^{‐\varphi \mu }\right)\left(e^{-y}y^{y}/y!\right){\left(e\mu /y\right)}^{\varphi \text{y}}},y=0,\\ \frac{\left(1‐\pi \right)\text{c}\left(\mu ,\varphi \right)\left(\varphi^{1/2}e^{‐\varphi \mu }\right)\left(e^{-y}y^{y}/y!\right){\left(e\mu /y\right)}^{\varphi \text{y}}}{1‐\sum_{y=4}^{\infty }\left(1‐\pi \right)c\left(\mu ,\varphi \right)\left(\varphi^{1/2}{\text{e}}^{‐\varphi \mu }\right)\left(e^{-y}y^{y}/y!\right){\left(e\mu /y\right)}^{\varphi y}},y=1,2,3. \end{array}\right. \end{array}$$

## 3. Results

In this study, 633 cardiovascular patients participated, of which 327 were male (51.7%). Mean age was 64.9 ± 6.68, 65.0 ± 6.51, 64.9 ± 6.71, and 66.4 ± 7.12 years for individuals with zero, one, two, and three coronary artery stenosis, respectively. Patients' BMI with zero, one, two, and three coronary artery stenosis was 26.7 ± 5.4, 26.6 ± 4.47, 27.5 ± 6.18, and 26.7 ± 5.47, respectively (Table 1). Baseline clinical features of patients—high sensitivity C reaction, smoking status, hypertension, diabetes, hyperlipidemia, history of cardiovascular diseases, and history of myocardial infarction—are reported by number of coronary artery stenosis in Table 1.

Truncated zero-inflated double Poisson model was performed on the number of coronary artery stenosis outcome. BMI and sex were significant predictors of the outcome in the count part of the model. Higher BMI (0.04; 95% CI: (0.01, 0.04), *p* = 0.011) and being female (0.19; 95% CI: (0.02, 0.36), *p* = 0.032) are found to be associated with higher number of coronary artery stenosis.

In regards to the results of logit part, BMI was the only significant factor. For every one-unit increase in BMI, the odds that the number of coronary artery stenosis would be a certain zero decrease by a factor of exp(−0.47) = 0.63 (*p* = 0.011). In other words, it is less likely that the number of coronary artery stenosis is zero as BMI increases.

Dispersion of the fitted outcome variable was investigated in the TZIDP model. The estimate of dispersion parameter (*ϕ*) was 0.23 (*p* < 0.001), suggesting that the estimated mean is less than the estimated variance in number of coronary artery stenosis outcome (Table 2).

To assess the validation of TZIDP model, goodness-of-fit statistics (including -2LogLikelihood and Akaike information criterion) were calculated and compared with alternative count models. The TZIDP model has shown the lowest goodness-of-fit statistics among all models (Table 3).

## 4. Discussion

In this study, we have established for the first time the truncated zero-inflated double Poisson model to characterize the effecting factors of the number of coronary artery stenosis.

In the present study, TZIDP, ZIDP, ZIP, ZINB, NB, and Poisson models were considered, and their performance was evaluated via goodness-of-fit measurements. The -2LL and AIC statistics indicate that TZIDP outperformed the other candidate models.

The descriptive results of the outcome variables show that the mean value (=1.7) is greater than the variance (=1.5), indicating underdispersion in the raw data. Although the difference ( = 0.2 = 1.7 − 1.5) is not significant, the double Poisson model was conducted. Once the TZIDP model is fit, the estimation of the dispersion parameter is in favor of overdispersion (*ϕ* = 0.23 < 1), suggesting that the estimated mean is less than the estimated variance in the fitted number of coronary artery stenosis. The advantage of using double Poisson model can be noted in this case, where there is no clear and strong evidence of under- or overdispersion in the observed data. The underlying assumption of traditional statistical distributions such as Poisson (equidispersion assumption) and negative binomial (over-dispersion assumption) models may not be tenable on the observed data before conducting the models. Under extreme cases, where the underdispersion scenario is obvious in the raw data, the above models may even encounter some convergence issues. Double Poisson model, on the other hand, has a dispersion parameter which makes the distribution more flexible to handle both over- and underdispersion scenarios. When designing the statistical analysis plan for a prospective study, it is not uncommon to have limited information about the expected distribution of a count variable whether over- or underdispersed. Double Poisson could be a smart choice in such situation which can offer flexibility around the dispersion parameter. Nevertheless, the nonlinear link function (mean of TZINB model is a nonlinear function of the model parameters) and the nonlinear relationship between dispersion parameter and mean and variance parameters could also explain the above result [23–25].

This literature shows that the zero-inflated models perform a better fit in the presence of excess zeros in the outcome. Using similar approach, various models have been discussed in this study to investigate the performance of conventional count models (ZIP vs. Poisson; ZINB vs. NB). In the presence of excess zeros, zero-inflated models are commonly used in literature. In this study, the goodness-of-fit measurements of ZI models are significantly lower than the non-ZI corresponding models, which is an expected finding. Zero-inflated regression models, by considering different probability functions for zeros and positive counts, would result in a less biased predicted values in compared to the observed values for the outcome. This has been also shown in literature [10, 13, 14].

The right truncation method is applied in this study as the outcome variable cannot take values > 3 due to theoretical range being 0, 1, 2, and 3. Without truncation, there will be predicted probabilities for the values out of the meaningful clinical range. This is a critical point which should not be ignored. Also, there is a significant improvement in the performance fit once right truncation model is applied. This is an expected result as the probabilities will be limited to the truncated range of the outcome values, which makes the predicted values to be closer to the observed values, and no prediction for the values out of the theoretical range will be calculated. Such improvement in the model fit with right truncation is also shown in literature [13, 26, 27].

In this study, the TZIDP model outperformed the alternative models based on the goodness-of-fit statistics, dealing with the excess zeros and right-truncated data with no underlying assumption about the outcome dispersion, i.e., TZIDP can handle dual data anomalies of excess zeros and right-truncated data in a count response variable where there is not a clear evidence of under- or overdispersion. Similar methodological ideas have been also reported in literature where there was some initial signals of overdispersion in the raw data [27–29].

It should be also noted that TZIDP is a complex model with many parameters. As a result, interpretations should be made with caution, and the estimates of the “count part” and the “logit part” of the model should be consistent for the same variable. For example, higher BMI in Table 3 is shown to be associated with higher number of coronary artery stenosis (count part) and lower likelihood of coronary artery stenosis being zero (logit part), which is consistent. Furthermore, the proposed model is able to improve the model fit significantly (Table 2); hence, it would be preferable in compared to the alternative models, aside from model complexity.

According to the fact that the number of coronary artery stenosis is zero in most patients, the proposed statistical can be an alternative approach to addressee both excess zeros and dispersion problems simultaneously for patients with coronary artery stenosis. The most important clinically relevant finding was that BMI and sex were significant predictors of the number of coronary artery stenosis in count part of the truncated zero-inflated double Poisson model, and BMI was the only significant predictor in logit part of the model.

Based on our findings, BMI is associated with the number of involved vessels which is consistent with some previous studies results. Indeed, our research confirmed other observations which considered BMI as an independent predictor in coronary endothelial dysfunction in patients with coronary artery disease [30, 31]. However, this finding is contrary to number of previous studies which have suggested that BMI was not an independent factor of coronary artery disease or severity on multivariate stepwise linear regression analysis anymore [32, 33]. This inconsistency might be due to the fact that our cohort is biased towards sever cardiovascular cases as well as elderly patients.

Several investigations have been previously reported gender differences in the distribution of risk factors of the number of coronary artery stenosis. In spite of differences between researches, our findings are consistent with previous reports [34, 35]. Our study showed that the number of coronary artery stenosis in women was 1.2 times more than men (*p* = 0.032). Due to the misperception of the protection against cardiovascular disease in females, the risk of heart disease is often underestimated in female group. As a result, aggressive treatment is less common on women rather than men in clinical trials, while the results of some studies have demonstrated that the number of coronary arteries involved was higher in men than women [36]. This result may be explained by the principle that the risk of coronary artery stenosis increases with age. Due to the effect of sex hormone function, women before menopause age are protected against coronary artery disease [37]. However, our results did not presume that age has a direct impact on the number of involved coronary arteries. Such contradiction in the impact of age could be due to the inclusion criteria of the current study where the intention was on elderly patients (>55 years old).

This study did not find a significant correlation between hs-CRP and coronary artery stenosis. Similar results did not find any association between CRP levels and angiographic extent score [38, 39]. These results reflect the finding of a review which evaluated the prognostic value of CRP in coronary artery disease. It was concluded that there were different biases in 83 previous studies, and the relationship between hs-CRP and prognosis is not strong [40].

Our outcome showed no significant correlation between diabetes mellitus and number of involved vessels (according to the classification in one, two and three vessel), but there was a probable considerable difference if it was evaluated based on one vessel and more than one vessel [33]. Other studies have been established that diabetics are more prone to multivessel coronary disease [41].

Concerning the amount of blood pressure, no statistically significant relationship between hypertension and the number of involved vessels was asserted. A positive relationship was reported in many studies [42, 43]. In spite of proved relation among hypertension, atherosclerosis, and coronary artery disease, other studies documented no significant association between hypertension and number of involved vessels. It should not be ignored that the focus of the current study is on severe cardiovascular elderly patients which might result in slightly different conclusion from the literature.

Angiography only shows lumen vessels and not the cross-sectional vessel wall morphology of vessel. Myocardial infarction usually is a consequence of angiographically nonobstructive lesions. This reality can explain why our results showed no significant relation between history of myocardial infarction and number of involved vessels [43].

## 5. Conclusion

The strength of this study was the novel methodology. As most patients had no coronary artery stenosis and number of involved vessels is limited to ≤3, the proposed model outperformed the conventional statistical methods. Potential limitation of the current study is the small sample size (single center study over <2 years of data collection) and the study design in terms of the eligibility criteria which limits the study population to severe cardiovascular elderly patients. Further investigations are required in larger studies, and the results could be validated in external cohorts of patients. Using the TZIDP model—as an alternative model—is advised to study the risk factors of number of involved vessels of coronary artery stenosis.

## Figures and Tables

**Table 1:** Demographic variables and baseline clinical features.

Variable	Number of coronary artery stenosis^∗^			
	0	1	2	3
	(*n* = 157)	(*n* = 104)	(*n* = 134)	(*n* = 238)
Age	64.9 ± 6.68	65.0 ± 6.51	64.9 ± 6.71	66.4 ± 7.12
Body mass index	26.7 ± 5.4	26.6 ± 4.47	27.5 ± 6.18	26.7 ± 5.47
High sensitivity C reactive protein	5.0 ± 5.36	7.0 ± 1.00	7.1 ± 9.03	6.8 ± 7.53
Gender (female)	109 (69.4)	46 (44.2)	60 (44.8)	91 (38.2)
History of smoking	44 (28.0)	41 (39.4)	47 (35.1)	83 (34.9)
Hypertension history	80 (51.0)	50 (48.1)	63 (47.0)	126 (52.9)
Diabetic history	43 (27.4)	38 (36.9)	44 (33.1)	97 (40.9)
Hyperlipidemia history	56 (35.7)	40 (38.5)	54 (40.3)	95 (39.9)
Cardiovascular diseases history	78 (49.7)	49 (47.1)	48 (35.8)	102 (42.9)
Myocardial infarction history	10 (6.8)	16 (16.5)	26 (20.6)	46 (20.3)

^∗^Mean ± standard deviation for continuous variables; frequency (%) for categorical variables.

**Table 2:** Parameter estimates using truncated zero-inflated double Poisson.

Parameter	Estimate	95% confidence interval	*p* value
Count part			
Body mass index	0.037	(0.01, 0.06)	0.011
Age (year)	-0.0005	(-0.017, 0.016)	0.956
Hypertension history	-0.047	(-0.497, 0.4)	0.837
Diabetic history	0.041	(-0.739, 0.821)	0.916
Gender (female)	0.19	(0.02, 0.36)	0.032
Myocardial infarction history	0.15	(-0.08, 0.38)	0.228
High sensitivity C reactive protein	0.011	(-0.001, 0.023)	0.086
Logit part			
Body mass index	-0.47	(-0.82, -0.12)	0.011
Age (year)	0.03	(-0.20, 0.26)	0.801
Hypertension history	0.57	(-4.90, 6.04)	0.837
Diabetic history	0.62	(-9.71, 10.95)	0.905
Dispersion (*ϕ*)	0.23	(0.09, 0.37)	<0.001

**Table 3:** Goodness-of-fit measurements of regression models.

Model	Goodness-of-fit statistics	
	−2LL	AIC
Truncated zero-inflated double Poisson	1522.4	1550.4
Zero-inflated double Poisson	1734.8	1762.8
Zero-inflated Poisson regression	1850.2	1876
Zero-inflated negative binomial regression	1850.2	1876
Negative binomial regression	1865.7	1882
Poisson regression	1865.7	1882

AIC: Akaike Information Criterion; −2LL: −2LogLikelihood.

## Data Availability

All data and materials are available from the corresponding author upon reasonable request.
